# Evaluation of Silk Fibroin-RGD-Stem Cell Factor Scaffold Effect on Adhesion, Migration, and Proliferation of Stem Cells of Apical Papilla

**DOI:** 10.1155/2021/6612324

**Published:** 2021-05-10

**Authors:** Jie Wei, Xiao-Qiang Sun, Ben-Xiang Hou

**Affiliations:** ^1^Department of Endodontics and Operative Dentistry, Capital Medical University School of Stomatology, Beijing/100050, China; ^2^Department of Stomatology, Peking University International Hospital, Beijing/102206, China

## Abstract

This study explored the effects of a silk fibroin-RGD-stem cell factor (SF-RGD-SCF) scaffold on the migration, proliferation, and attachment of stem cells of apical papilla (SCAPs). SF, SF-RGD, SF-SCF, and SF-RGD-SCF scaffolds were prepared, and laser confocal microscopy was used to observe the adhesion and growth status of SCAPs on the scaffolds. Furthermore, the numbers of SCAPs on the scaffolds were counted by a digestion counting method to evaluate their proliferation. Cells on the SF-RGD-SCF scaffold proliferated more than those on the other scaffolds and showed a more obvious tendency to migrate to the scaffold's deep porous structure after 7 d seeding. Live/dead cell staining results showed that almost all the adhered cells were alive after 7 d. Furthermore, cell counting showed that the number of cells on the SF-RGD-SCF scaffold was highest after both 1 and 7 d (*P* < 0.05). Thus, the SF-RGD-SCF composite is biocompatible and promotes the migration, adhesion, and proliferation of SCAPs, making it of potential use as a scaffold for cell-homing pulp regeneration.

## 1. Introduction

Root canal treatment is currently the most common method for addressing irreversible pulpitis and periapical periodontitis of teeth. Although teeth can survive this treatment, the resistance and anti-infection ability of the residual dentin are greatly reduced due to poor nutrition supply [1]. When immature permanent teeth are deprived of dental pulp due to caries, trauma, and/or abnormal development, they cannot form dentin in the root area, which makes the root dentin wall too thin to perform its functions [2]. These changes in anatomical and functional conditions result in the failure of pulp treatment for immature permanent teeth and an increased incidence of tooth fracture, which reduces tooth survival rate [3–5]. Accordingly, replacing infected and/or necrotic dental pulp using a system that enables the regeneration of dental pulp is an attractive strategy for the future treatment of dental pulp diseases. Such a treatment strategy would extend the service life of the affected teeth and improve the living quality of patients [6].

Pulp regeneration involves the reconstruction of the pulp-dentin complex, restoring the physiological function of the pulp. This kind of tissue engineering requires three major elements: stem cells, growth factors, and scaffold materials [7].

There are two major technologies in dental pulp engineering research. The first is a cell-based approach for dental pulp tissue regeneration. This technology requires the introduction of exogenous stem cells to root canals, also termed “stem cell translation.” The second is a cell-free approach. This technology does not need the introduction of exogenous stem cells. Instead, it involves endogenous stem cells homing into the pulp regeneration site, also called “cell homing” [8]. Cell-based dental pulp tissue engineering technology requires stem cell transplantation, and this technology is complex, highly sensitive, and high cost. However, cell homing is based on chemokines recruiting endogenous stem cells, avoiding the cell processing steps required for cell transplantation and making full use of the patient's own stem cells, which reduces operation difficulty and risk and is more easily applied clinically [9].

For the cell homing technique, the choice of appropriate signaling molecules that induce apical papilla stem cells to migrate to the regeneration site while maintaining or maximizing their differentiation potential is crucial [10]. Such signaling molecules, including growth factors, cytokines, and hormones, are biological cues that activate regeneration processes [9]. As a representative signaling agent, stem cell factor (SCF) has been demonstrated to have positive effects on the migration of bone marrow mesenchymal stem cells [11].

There are also certain requirements for the scaffold materials used in cell-homing treatments. The scaffold needs to promote the adhesion, infiltration, vascularization, and cell differentiation of recruited cells and provide a favorable microenvironment for the regenerated dental pulp [12]. Furthermore, an ideal tissue-engineering scaffold should be biodegradable, allowing it to be ultimately replaced by the regenerating tissue [13].

Silk fibroin (SF) is mainly composed of glycine, serine, and alanine in a highly repetitive polypeptide chain. It is a natural biological material that exhibits slow degradation, good biocompatibility, low immunogenicity, low toxicity, and good mechanical properties [14], and it can be processed into a variety of forms such as films, gels, and stents. Accordingly, there is extensive tissue-engineering research on the use of silk materials as scaffolds for bone, cartilage, ligament, connective tissue, and skin [15, 16]. Furthermore, RGD peptide (arginine-glycine-aspartic acid), a polypeptide derived from fibronectin, is widely used on the surface of synthetic materials to facilitate cell adhesion [17–20].

The adhesion, migration, and proliferation of stem cells of apical papilla (SCAPs) on SCF-loaded, RGD-conjugated SF (SF-RGD-SCF) scaffold materials have not been reported to date. Accordingly, in this study, we have tested the hypothesis that SF-RGD-SCF scaffolds can promote SCAP adhesion, migration, and proliferation.

## 2. Materials and Methods

### 2.1. Preparation of SF Scaffolds

SF protein was isolated from silkworm (*Bombyx mori*) cocoons by a standard isolation procedure [21]. Three-dimensional (3D) sponge SF scaffolds were prepared by freeze drying. Briefly, 3 mL drops of a SF solution (9 wt%) were placed in the wells of a 24-well plate and cooled at -10°C overnight. The scaffolds were then freeze dried for 24 h at -80°C and soaked in ethanol for 24 h to promote cross-linking. Finally, the material was dried at room temperature to obtain a porous 3D fibroin scaffold. The structure of the SF scaffold was confirmed using scanning electron microscopy (SEM, Quanta 200FEG FEI, USA).

### 2.2. Conjugating RGD Polypeptide to the Scaffolds

The prepared SF scaffolds were immersed in phosphate buffered saline (PBS, Gibco, Grand Island, NY) for 30 min then soaked in a 1-(3-dimethylaminopropyl)-3-ethyl carbodiimine hydrochloride (Shanghai Yuanye Bio-Technology Company, Shanghai, China) and *N*-hydroxy succinimide (Shanghai Yuanye Bio-Technology Company, Shanghai, China) mixture to react for 30 min. They were then rinsed thoroughly with PBS to wash off the remaining chemical reagents. Finally, 0.5 mL RGD polypeptide (GRGDSPC, NJPeptide, Jiangsu, China) at 0.1 mg/mL in PBS was reacted with SF scaffolds for 2 h to obtain SF-RGD scaffolds.

### 2.3. Sterilization and Preincubation

Before loading SCF into the scaffolds, they were sterilized in ethanol (75%) for 1 h then exposed to UV irradiation for 2 h after removing the residual ethanol with PBS. After sterilization, the scaffolds were immersed into *α*-minimum essential medium (*α*-MEM, Gibco, Grand Island, NY) containing 15% fetal bovine serum (FBS, Gibco, Grand Island, NY) to preincubate for 2 h at 37°C. All remaining operations were completed on a clean bench.

### 2.4. Loading of SCF into the Scaffolds

A Recombinant Human SCF/c-kit Ligand (R&D Systems, Minneapolis, MN, USA) reagent mixture was made into a 10 *μ*g/mL solution according to the manufacturer's instruction. On a clean bench, sterile blotting paper was used to dry the scaffolds; then, 6 *μ*L SCF solution (10 *μ*g/mL) was dropped into the center of the dried scaffolds. The 24-well plates containing the materials were then placed at room temperature for 1 h to allow the adhesion of SCF to the scaffolds [21].

### 2.5. Isolation, Characterization, and Expansion of SCAPs

Apical papilla tissues were obtained from normal human impacted third molars (18–24 years of age) with informed consent and under Dental Clinic guidelines as approved by the Ethics Research Committee of Capital Medical University of Medical Sciences (reference no. CMUSH-IRB-KJ-PJ-2019-02F). Two teeth were used in this study.

Apical papilla tissue was gently separated and cut into small pieces from the root. For digestion, apical papilla pieces were placed into a mixture of collagenase type I (Sigma-Aldrich, St Louis, MO) solution (6 mg/mL) and dispase (Sigma-Aldrich, St Louis, MO) solution (8 mg/mL) for 1 h at 37°C. The released single cells were grown in a culture dish (60 mm × 15 mm) with 5 mL *α*-MEM containing 20% FBS, 1% penicillin-streptomycin (Gibco, Grand Island, NY), and 1% L-glutamine (Gibco, Grand Island, NY). The primary culture cells were digested with 0.25% trypsin (Gibco, Grand Island, NY) and passaged till monolayer cells spread to more than 80% of the bottom of the culture dish, and the passaged cells were then grown in a culture dish (100 mm × 20 mm) with 10 mL *α*-MEM containing 15% FBS, 1% penicillin-streptomycin, and 1% L-glutamine. SCAPs were incubated at 37°C under 5% CO_2_. SCAPs between the 3rd and 5th passages were used throughout the study.

The *in vitro* differentiation of SCAPs into osteogenic and adipogenic lineages was evaluated by induction with osteogenic (15% FBS, 1% penicillin-streptomycin, 1% L-glutamine, 1% ascorbic acid, 1% *β*-glycerophosphate, and 1% dexamethasone) and adipogenic media (Gibco, Grand Island, NY) for 21 d and then Alizarin Red (Beyotime Institute of Biotechnology, Jiangsu, China) and Oil Red O staining (Beyotime Institute of Biotechnology, Jiangsu, China) to identify mineralization and formation of neutral lipids [22].

### 2.6. Cell Seeding

After the scaffolds were incubated under standard cell culture conditions (37°C, 5% CO_2_) for 2 h, 100 *μ*L of cell suspension containing 5 × 10^5^ SCAPs was dropped onto the scaffold. After incubating the cell-loaded scaffold for 4 h under standard cell culture conditions, 500 *μ*L culture medium (*α*-MEM containing 15% FBS, 1% penicillin-streptomycin, 1% L-glutamine) was added to the plate containing cell-laden scaffold and exchanged every three days [23, 24].

### 2.7. Transwell Migration Assay

SCF solutions without a scaffold and SF, SF-SCF, and SF-RGD-SCF scaffolds were cultured in the lower compartment of 24-well plates, whereas SCAPs were grown on a permeable transwell support insert (Corning Inc. Foundation, Tewksbury, MA). An SF scaffold served as a negative control, and a 600 *μ*L solution with 100 ng/mL SCF and culture medium (*α*-MEM containing 15% FBS, 1% penicillin-streptomycin, 1% L-glutamine) served as a positive control.

The 24-well plates with transwell inserts were incubated at 37°C and 5% CO_2_. The transwell insert was carefully removed after 24 h incubation, and the cells that had not migrated through the pores were gently removed with cotton swabs.

Cells on the lower side of the insert filter were fixed in 4% paraformaldehyde for 1 h and incubated with 0.1% 2-(2-[4-(1,1,3,3-Tetramethylbutyl)phenoxy]ethoxy)eth (Triton X-100, Beyotime Institute of Biotechnology, Jiangsu, China) at room temperature for 30 min. Then, the cells were incubated with 40,6-diamidino-2-phenylindole (DAPI, Beyotime Institute of Biotechnology, Jiangsu, China), for 15 min. Translated cells were observed under a laser confocal microscope (Leica, Germany), and the cell numbers of nine microscopic vision fields for each group were counted and analyzed.

### 2.8. Cell Proliferation

Cell-loaded scaffolds were cultured in 24-well plates for 1 or 7 d. Then, the cells on the scaffolds were digested with 0.25% trypsin and suspended in *α*-MEM. An automatic cell counter (TC10TM, Bio-Rad Laboratories, USA) was used to count the number of cells on each scaffold.

### 2.9. Immunofluorescence

For immunohistochemical fluorescence analysis, cell-loaded scaffolds were cultured in 24-well plates for 1 or 7 d and fixed in 4% paraformaldehyde. The cell-loaded scaffolds were washed three times before being incubated with 0.1% Triton X-100 at room temperature for 30 min and then incubated with 5% bovine serum albumin (BSA, Gibco, Grand Island, NY) at 37°C for 1 h. The cell-loaded scaffolds were washed three times before being incubated with Rhodamine Phalloidin (Beyotime Institute of Biotechnology, Jiangsu, China) at 1 : 200 dilution overnight at 4°C and then incubated with DAPI for 15 min. Immunoreactivity was assessed using a laser confocal microscope.

### 2.10. Live/Dead Assay

After 7 days of culture, the cell-containing scaffolds were removed and placed in a new 24-well plate. The scaffolds were washed gently with PBS 3 times for 5 min each time. A live/dead staining kit (Thermo Fisher Scientific, Pittsburgh, PA) was removed from the refrigerator in advance and brought to room temperature. The reagent was then diluted with PBS to a working concentration (2 *μ*g/mL calcitonin and 4 *μ*g/mL bromoethorphine dimer). Each scaffold was added to 0.5 mL of the working reagent and soaked for 40 min at room temperature. PBS was used to wash the scaffolds three times, and 0.5 mL 4% paraformaldehyde solution was used to fix the cells for 1 h. Then, PBS was used to wash the cells again three times. Finally, aseptic filter paper was used to dry the scaffolds, and the sheet was sealed. The cells were then observed under a laser confocal microscope.

### 2.11. Statistical Analysis

Data are presented as mean ± standard deviation (*n* ≥ 3 per group) in this paper. Statistical significance was determined by paired samples *t*-test using the SPSS 17.0 software.

## 3. Results

### 3.1. Characterization of SF Scaffold

The SF scaffolds prepared in this study were circular with a diameter of 1.5 cm and a thickness of ~3 mm. The dried SF scaffolds were hard and brittle but turned elastic and plastic upon absorbing water. Using SEM, the SF scaffolds were observed to have 3D porous structures with uniform pore diameters of ~100 *μ*m (Figure 1).

### 3.2. Characterization of SCAPs

The primary cells grew out from the tissue block after 5 d culturing, showing plastic adherence and exhibiting spindle shapes (Figure 2(a), A'). After 3 weeks osteogenic induction, extensive amounts of mineralized nodules were observed in the cultured cells (Figure 2(b)). A small number of lipid droplets were observed with oil red O staining after 3 weeks of adipogenic induction (Figure 2(c)).

### 3.3. Cell Migration

Transwell assay was performed to evaluate the effect of SCF on the migration capacity of SCAPs. The laser scanning confocal microscope images indicate that the migratory cells in the SCF, SF-SCF, and SF-RGD-SCF groups are significantly denser than those in the SF group (Figure 3). Groups having SCF show significantly promoted cell migration compared with the control group after 24 h cell seeding (*P* < 0.01) (Figure 4). Furthermore, there is no significant difference between the SCF, SF-SCF, and SF-RGD-SCF groups (Figure 4).

### 3.4. Cell Proliferation

After being cultured in different scaffolds for 1 or 7 d, the proliferation ratios of the SCAPs in the SF-SCF-RGD scaffolds are significantly higher than those of the control group at every time point (*P* < 0.05). However, there is no significant difference between the SF-RGD-SCF and SF-RGD groups. Furthermore, there is no significant difference between the SF-SCF and SF groups (Figure 5).

### 3.5. Cell Spread and Adhesion

The cells on the scaffolds were observed under a laser confocal microscope after 1 and 7 d culturing and immunofluorescence staining. SCAPs were observed to be spreading and adhering for all the scaffolds, with the cells on scaffolds with RGD spreading much better those without RGD. Furthermore, cells on the former adhere more strongly than those on the latter (Figures 6 and 7).

After 1 d culture, the cells on SF and SF-SCF scaffolds do not exhibit intercellular contact, whereas those on SF-RGD and SF-RGD-SCF are observed to have formed intercellular contacts (Figure 6).

After 7 d culture, all the scaffolds are covered with SCAPs, and all show intercellular contact (Figure 7). Furthermore, the cells on SF-SCF and SF-RGD-SCF scaffolds migrate deeper into the support structure than those on the SF and SF-RGD scaffolds (Figures 7(a3), 7(b3), 7(c3), and 7(d3)).

### 3.6. Cell Biocompatibility (Live/Dead Assay)

The results of live/dead assays show that all the scaffolds exhibit good cell biocompatibility for SCAPs. After 7 d culturing, most of the cells on the scaffolds are alive (Figure 8). The SF-RGD, SF-SCF, and SF-RGD-SCF scaffolds show more living cells than the SF group (Figures 8(a3), 8(b3), 8(c3), and 8(d3)). This result is in good agreement with the cell counting and adhesion results.

## 4. Discussion

Odontogenic stem cells include SCAPs, dental pulp stem cells (DPSCs), periodontal ligament stem cells, dental capsule stem cells, and stem cells from the pulp of deciduous teeth [7]. Among them, DPSCs and SCAPs are commonly used as seed cells for pulp regeneration, and SCAPs are more capable of proliferation and mineralization than DPSCs [25]. Huang et al. have reported that SCAPs can differentiate into odontoblast cells and form root dentin during root development as well as guiding pulp regeneration [26, 27]. Thus, SCAPs were chosen in our study to test the adhesion-, migration-, and proliferation-promoting abilities of the SF-RGD-SCF scaffold.

Cell homing is a normal physiological process related to posttraumatic healing in which stem cells enter the sterile root canal with the formation of supporting tissues such as blood vessels and nerves [28, 29]. Studies have shown that trauma or iatrogenic factors can separate the root tip area from the main tooth root, and the epithelial root sheath and apical papilla stem cells in the separated root tip area can continue to develop into a separate root tip structure [30]. Furthermore, the apical papilla has been proved to be active in the case of pulp necrosis [31]. These findings indicate that it is possible to use endogenous stem cells for pulp regeneration.

Cell homing has numerous advantages over the transplantation of cells into root canals, as such cells cannot form circulation and cause damage to root tips [32]. However, a remaining problem is that the number of mobilized and activated stem cells is typically too small to fill the damaged tissue for repair or regeneration [9]. Studies have found that cytokines, as key signaling molecules for cell homing, can mobilize endogenous stem cells and regulate the proliferation and differentiation of stem cells and progenitor cells [33, 34]. As one such cytokine, SCF was originally found in hematopoietic stem cells, which bind to c-kit receptors on the surface of hematopoietic stem cells and play a role in inducing the maturation of precursor hematopoietic stem cells. Furthermore, SCF/c-kit channel can induce cell proliferation and migration [12]. SCF/c-kit combination occurs on the surface of odontogenic stem cells, such as dental pulp stem cells, dental sac stem cells, and periodontal ligament stem cells, and SCF can promote the proliferation, migration, neovascularization, and collagen remodeling of dental pulp progenitor cells [35]. In our research, after being cultured in different scaffolds for 1 or 7 d, the proliferation ratios of the SCAPs in the SF-SCF-RGD scaffolds are the highest. However, our results find that SF-RGD and SF-RGD-SCF scaffolds have more cells than the other two groups after 1 d culturing, which may indicate that scaffolds with RGD can attach more cells in the early stage. We can get support from Hasenbein's research [36], which found that RGD can enhance the adhesion of fibroblasts and osteoblasts. In the meantime, after being cultured for 7 d, the number of SCAPs in the SF-SCF group is higher than the SF and SF-RGD group, which may remind us that SCF plays an important role increasing the number of SCAPs in the later stage. Our results are consistent with these previous findings. Further experimentations are needed to prove how the SF-RGD-SCF scaffold promote the adhesion and proliferation of SCAPs.

Stromal cell-derived factor-1 (SDF-1) is another cytokine commonly used for cell homing. SDF-1 promotes the migration of dental pulp stem cells, induces stem cell homing to canine teeth in dogs, and induces the proliferation and differentiation of dental-pulp-like tissues [37]. SDF-1 has been indicated to be related to angiogenesis and tumor formation, whereas no direct relationship between SCF and tumor growth has been demonstrated [38, 39]. In this aspect, SCF may be a better choice for cell homing treatment.

## 5. Conclusions

The SF-RGD-SCF scaffold developed in this study is biocompatible and could promote the migration, adhesion, and proliferation of SCAPs. It is potential to be used as a scaffold for cell-homing pulp regeneration.

## Figures and Tables

**Figure 1:** Microstructure of an SF scaffold. Under SEM, a 3D porous structure with uniform pores of ~100 *μ*m in diameter can be observed (640x, scale bar = 100 *μ*m).

**Figure 2:** Growth and differentiative capacity of SCAPs. (a) Primary SCAPs after 5 d culture (scale bar = 2 mm). (A') Primary SCAPs after 5 d culture (scale bar = 200 *μ*m). (b) Alizarin Red staining results showing the extent of osteogenesis (scale bar = 100 *μ*m). (c) Oil red staining showing the extent of adipogenesis (scale bar = 100 *μ*m).

**Figure 3:** The nuclei of migratory cells stained with Hoechst 33258: (a) SCF group; (b) SF-SCF group; (c) SF-RGD-SCF group; (d) SF group.

**Figure 4:** Migrated cell numbers (each vision field) for SCF, SF-SCF, SF-RGD-SCF, and SF groups. Data are means with SD error bars (*n* = 9). ^∗∗∗^*P* < 0.001 compared with the negative control (SF).

**Figure 5:** Cell numbers after 1 and 7 d cell seeding: (a) 1 d; (b) 7 d. Data are means with SD error bars in (*n* = 3). ^∗^*P* < 0.05, ^∗∗^*P* < 0.01, ^∗∗∗^*P* < 0.001.

**Figure 6:** Laser scanning confocal microscopy images of cells on scaffolds after 1 d seeding. Cell cytoskeletons were stained with Rhodamine Phalloidin (a1, b1, c1, d1). Cell nuclei were stained with Hoechst 33258 (a2, b2, c2, d2). Merged pictures of cell cytoskeletons and nuclei (a3, b3, c3, d3) (red arrows: cell cytoskeletons; yellow arrows: cell nuclei).

**Figure 7:** Laser scanning confocal microscopy images of cells on scaffolds after 7 d seeding. Cell cytoskeletons were stained with Rhodamine Phalloidin (a1, b1, c1, d1). Cell nuclei were stained with Hoechst 33258 (a2, b2, c2, d2). Merged pictures of cell cytoskeletons and nuclei (a3, b3, c3, d3) (red arrows: cell cytoskeletons; yellow arrows: cell nuclei).

**Figure 8:** Laser scanning confocal microscopy images showing live and dead cells after 7 d seeding. Live cells show as fluorescent green (a1, b1, c1, d1). Dead cells show as red (a2, b2, c2, d2). Merged pictures of live and dead cells (a3, b3, c3, d3) (white arrows: live cells; blue arrows: dead cells).

## Data Availability

(1) The (figures) data used to support the findings of this study are included within the article. (2) The (bar graphs) data used to support the findings of this study are included within the supplementary information files.
